RETRACTED

# Analysis of Herdsmen's Credit Behavior under the Identification Scheme of Emotional and Psychological State

**DOI:** 10.1155/2022/9288896

**Published:** 2022-10-06

**Authors:** Xinling Zhang, Huijie Huang, Liyang Zheng

**Affiliations:** ^1^College of Economics and Management, Inner Mongolia Agricultural University, Hohhot 010051, China; ^2^College of Humanity and Social Science, Inner Mongolia Agricultural University, Hohhot 010051, China

## Abstract

Herdsmen's access to credit funds plays an important supporting role in promoting the modern economic development of pastoral areas and broadening the channels for herders to increase their income. This paper studies the credit behavior of herdsmen from the perspective of emotional and psychological state identification to analyze the current credit behavior of herdsmen. Firstly, the internal mechanism of herdsmen's credit and emotional and psychological identification research content are analyzed. Secondly, a scheme of emotional and psychological state identification is proposed, and a corresponding survey of herdsmen is carried out according to the scheme. Finally, the Probit and Heckman models are introduced to analyze the credit behavior of herdsmen. The results show that herdsmen with high emotional and psychological scores strongly demand credit. They are likely to have access to credit and have a high level of credit. Herdsmen with low scores of emotional and psychological characteristics have low or no apparent demand for credit, and their credit availability is also low. The herdsmen with high emotional and psychological characteristics have a 71% higher probability of generating credit demand than herdsmen with low openness. Their likelihood of obtaining credit is also 33.47% higher than herdsmen with low emotional and psychological characteristics. They also have easy access to higher loan amounts. The results provide a reference for related research and analysis of herdsman's credit behavior and economic development.

## 1. Introduction

Credit is an important policy tool for addressing poverty in pastoral areas. It has played an important role in developing “agriculture, rural areas, and farmers” for a long time. The “separation of rural land ownership, contract rights, and management rights” and “socialized services” have been continuously promoted. Land and labor constraints are eased through the transformation of capital factors [1]. Therefore, the financial constraints are prominent, and high requirements are placed on the precision and flexibility of rural credit products and services [2]. In addition, the enthusiasm of herdsmen for pasture circulation is high, driven by the need to expand the scale and ensure the sense of fatness [3]. The pasture transfer market is increasingly active. The interactive logic of grassland circulation and credit is an important prerequisite for studying the relationship between grassland circulation and the coordinated development of financial markets in agricultural and pastoral areas. However, the impact of land on credit is by no means limited to owned land. Numerous studies have shown that the transfer of non-all arable land also significantly impacts farmers' access to credit in formal financial institutions. Farmland transfer can effectively alleviate demand-based credit constraints. The transfer of farmland makes farmers have a demand for agricultural credit. The need for credit also increases with the transfer of agricultural land [4]. Overall, farmland transfers can increase farmers' access to credit. However, this opportunity is not equal, widening the gap between rich and poor farmers in access to credit [5]. The transfer of farmland cannot relieve farmers' credit constraints but will reduce the loan intensity, resulting in severe credit constraints [6].

RETRACTED

Besides, information science can be organically combined with the research paradigm of psychology with the rapid development of modern information science and technology such as intelligent wearable sensing technology, virtual reality technology, computer network technology, data mining technology, and artificial intelligence technology. Traditional psychometric research methods and tools can be effectively improved [7]. Intelligent measurement methods can bring comprehensive and rich multisource data to psychological measurement, so they are gradually applied in psychological research [8]. The key technologies of emotional and psychological state recognition based on multisource information fusion are studied under traditional research methods. It can help identify individuals' psychological characteristics such as intelligence, personality, and psychological health differences to determine their relative strengths and weaknesses. This will provide a quantitative basis for teaching students according to their aptitude and using their talents best [9]. In analyzing herdsman's credit behavior, the individual differences between herdsmen's credit behavior are obtained by analyzing and identifying their emotional and psychological states. Credit additional measures are implemented according to herdsmen's differences in credit behavior [10].

Researchers have also conducted a lot of studies in the corresponding field. Pang et al. [11] proposed a herdsman credit quality assessment method based on an extreme learning machine, fuzzy c-means algorithm, and confusion matrix calculation through the weight of the evidence evaluation method and the calculation of information value. They built borrower credit scoring models by screening credit rating indicators. They also constructed equations to determine the Probability of Default (PD) and Loss Given Default (LGD). They collected sample data of 7,706 loan borrowers from the Internet. The borrower's credit score, PD for each type of borrower, and LGD were calculated. The repayment status of the borrower was analyzed. The experimental results showed that the overall accuracy of the credit scoring model was 98.5%, including 98.9% for nondefault samples and 88.3% for default samples. Lee and Lee [12] used six credit attitude variables to construct a comprehensive index variable of credit attitude. They used aggregated data from the 2010 and 2013 Consumer Finance Surveys released by the Board of Governors of the Federal Reserve System. The analysis results showed that the credit attitude index had a positive impact on payment behavior. Households with more favorable attitudes toward nonessential credit use were likelier to have outstanding credit card balances, irregular payment habits, and recurring charges. Bian et al. [13] studied the black box of bank credit smoothing behavior. The sample was 128 Chinese banks from 2007 to 2014. Politically connected banks were identified by their chairman's government experience. It was found that the lending behavior of non-state-owned banks with political ties was less procyclical than that of non-state-owned banks with no political ties. In addition, there was no heterogeneity in the lending behavior of state-owned banks with political ties and state-owned banks without political ties. At present, the research and application of emotional and psychological state recognition technology in behavior management are still in infancy. In particular, there are few studies on the application and innovative research in analyzing herdsman behavior.

RETRACTED

This paper is organized as follows. Firstly, the research background and significance of this subject are introduced, and the research process and research status related to this subject are analyzed. Then, the research on the universal intelligent psychological evaluation system is carried out. The psychological assessment system and technical architecture are analyzed and designed from the overall requirements of the system. Finally, research on the method of mental state identification based on multisource information fusion is conducted. In addition, three multisource information fusion strategies for the data layer, feature layer, and decision layer fusion are comprehensively compared. Then, a *P* value evaluation method of emotional and psychological state based on feature layer fusion and an emotional and psychological state recognition method based on decision layer fusion are proposed.

The innovation and contribution are the research on the key psychometric technology of multisource information fusion based on the intersection of psychology and information science. A set of the universal intelligent psychological evaluation systems is analyzed, designed, and implemented based on the traditional psychometric research paradigm, which provides a reference for different fields and institutions to realize the intelligentization of psychometric work. Meanwhile, an emotional and psychological state recognition method based on feature layer fusion and decision layer fusion is proposed. Finally, the microhouseholds of 200 herdsmen in three autonomous banners in XX district are investigated. The influence of herdsman's credit access is analyzed using herdsman's emotional and psychological state.

## 2. Methods

### 2.1. Analysis of Emotional and Psychological State Recognition Technology

Studies have indicated that changes in human emotional states can cause a combination of changes in physiology, facial expressions, speech, and body posture. The signals of these changes can independently represent a particular emotional stat. The multisource information fusion calculation method for emotional and psychological recognition can fully use the complementarity and redundancy between homogeneous or heterogeneous data, thereby improving the accuracy of emotional and psychological recognition. Therefore, the psychological characteristics to be measured are thoroughly and objectively displayed. Many scholars have gradually formed a good development trend [14]. The general steps of the calculation process of emotional and psychological recognition based on multisource information fusion are shown in Figure 1.

From Figure 1, the general steps of the calculation process of emotional and psychological recognition based on multisource information fusion are as follows. The first is to choose an emotional induction method. The HCI system completes specific tasks according to the audio-visual materials and selects the appropriate emotional induction method according to the obtained results. The second is to collect physiological signals. Transform according to different information fed back by multiple sensors. Besides, appropriate signal values are collected. The third is signal preprocessing. The collected physiological signals are first processed into frames, and extreme values are removed and smoothed according to different filter values. Finally, the output signal values are detected by characteristic waveform points. The fourth is emotional feature extraction. It mainly extracts time-domain features, frequency domain features, time-frequency domain features, and nonlinear features in signal values. The fifth is feature fusion. The collected features are fused. The sixth is to divide the dataset. The processed data values are divided into training and sample sets. The seventh is to classify the sample dataset and the internal data of the training set, and the recognized emotional and psychological state is output [15].

RETRACTED

The data feature layer fusion is further analyzed. Feature layer fusion refers to the feature extraction of multisource signals, respectively. Then, these multimodal features are formed into a joint feature vector according to a fusion algorithm. This vector is fed into the same classifier to output the recognition result [16]. Physiological state recognition is taken as an example. The general process of feature layer fusion is shown in Figure 2.

From Figure 1, the feature layer fusion process needs to extract information about people's psychological states through multiple sensors. Feature extraction is performed after the information source is obtained. The extracted features are fused, and the final recognition result is output after classification by the classifier. In emotional and psychological recognition, existing feature layer fusion methods consist of principal component analysis, linear discriminant analysis, kernel matrix fusion, and genetic algorithm. The feature layer fusion method effectively utilizes the correlation and complementarity between different features but ignores the differences between features. It also requires high synchronization between various modal features. However, it improves the classification accuracy of the classifier and facilitates real-time processing [17].

Decision layer fusion refers to the feature extraction of multisource signals, respectively. Then, they are input into the respective classifiers to get the classification results. The classification results are fused according to specific criteria to output the final recognition result [18]. Physiological state recognition is taken as an example. The general process of decision-level fusion is demonstrated in Figure 3.

In Figure 3, different sensors are located at different positions on the human body. Sensor 1 is located on the subject's head, sensor 2 is located on the subject's upper limb, and sensor *n* is located on the subject's lower limb. From Figure 3, the fusion process of the decision-making layer needs to extract information from people's psychological states through multiple sensors. Feature extraction is performed after the information source is obtained. The classifier classifies the extracted features, and the output results are fused for decision-making to get the recognition results [19].

RETRACTED

Feature layer fusion and decision layer fusion strategies are widely used in practice, so an emotional and psychological state recognition method based on the fusion of these two levels is proposed here [20].

### 2.2. Analysis of the Current Situation of Herdsmen's Credit

Sufficient economic resources are the core factor for individual development and even the realization of freedom. Still, the current economic and social credit constraints are severe, which limits the herdsmen's pursuit of freedom. Therefore, enhancing credit availability for herdsmen has always been a research focus in the financial field. The government has taken a series of measures to increase the monetary supply of herdsmen to deepen the development of herdsmen's financial inclusion, such as guiding financial institutions to carry out small loan business, giving herdsmen financial services tax incentives, and relaxing the access threshold of financial institutions [21]. However, although these measures have eased the constraints on credit supply, they have not yet achieved ideal results in improving the credit availability to herders. The reason is that the credit availability of herdsmen is not only related to the credit rationing of financial institutions but also influenced by herdsmen's characteristics, especially herdsmen's psychological characteristics [22].  Figure 4 reveals the effect of herdsman's emotional and psychological characteristics on herdsman's credit demand.

From Figure 4, emotional and psychological characteristics directly affect risk appetite, affecting credit demand [23]. Using credit is a risky act. Individuals with different emotional and psychological characteristics have other risk preferences and abilities to bear, so their credit needs differ. Second, the emotional and psychological characteristics will affect the individual's production and operation mode, especially the entrepreneurial choice, and indirectly affect their credit demand. Finally, the emotional and psychological characteristics take human capital a role, especially the educational level, which indirectly impacts the credit demand of herdsmen. Education level is widely recognized as a critical variable affecting herdsmen's demand for credit. There are three possible pathways for how emotional-psychological characteristics affect herdsmen's access to formal credit. The first is the social network that affects herdsmen. The second is to influence the formal credit availability of farmers by affecting the guarantee capacity possessed by herdsmen [24]. The lack of legally eligible collateral makes secured loans the primary way for farmers to obtain formal credit. The third is that different personality characteristics make farmers' information transmission ability and information recognizability significantly different, affecting their formal credit availability [25–28].

RETRACTED

### 2.3. Emotional and Psychological State *P* Value Evaluation Method Based on Feature Layer Fusion

The evaluation method of the emotional and psychological state *P* value based on the fusion of the feature layer is as follows according to the questioner's choice of the answer to the test question, the expression, and the fusion characteristics of various physiological and psychological signals.

1. Assuming that the scale used in the intelligent question and answer session contains *N* factors, the question and answer records of the subjects are obtained after the intelligent question and answer session. Lie detection is combined with facial expression recognition when the subjects answer questions. If the expression conforms to the preset, the answer to the question is recorded as valid. The answer records are calculated according to the quantitative scoring rules of the scale to which the item belongs. The fractional value of *N* factors is obtained, denoted as a column vector *A*, as shown in

(1) $$\begin{array}{c} \text{A}=\left[\begin{array}{c} n_{1}\\ n_{2}\\ \cdots \\ n_{N} \end{array}\right]. \end{array}$$

(2) Assuming that the period when the animation game session induces a particular emotion is *t*, the facial expression and *M*-type physiological data of the subjects within *t* are collected. The original facial expression data during this period is denoted as *E*. The feature extraction rule *f* is used to extract the expression feature value for the expression image with the most significant proportion of expressions in the original data, denoted as *f*(*E*). The *M*-type original physiological signals are represented as *B*_1_, *B*_2_, ⋯*B*_*M*_. The feature extraction algorithm *f*_*i*_ corresponding to each physiological signal is used. Feature extraction is performed on *B*_1_, *B*_2_, ⋯*B*_*M*_ to extract the eigenvalues of *M*-type physiological signals. The expression and physiological signal eigenvalues are concatenated into a joint eigenvector *B*
(3) The combined eigenvectors obtained from the three psychometric steps are weighted and fused to get the fusion eigenvector *P*. It is obtained according to

(2) $$\begin{array}{c} P=\alpha \cdot A+\beta \cdot B,\\ P=\alpha \cdot \left[\begin{array}{c} n_{1}\\ n_{2}\\ \cdots \\ n_{N}\\ 0 \end{array}\right]+\beta \cdot \left[\begin{array}{c} f\left(E\right)\\ f_{1}\left(B_{1}\right)\\ f_{2}\left(B_{2}\right)\\ \cdots \\ f_{M}\left(B_{M}\right) \end{array}\right],\\ B=\left[\begin{array}{c} f\left(E\right)\\ f_{1}\left(B_{1}\right)\\ f_{2}\left(B_{2}\right)\\ \cdots \\ f_{M}\left(B_{M}\right) \end{array}\right]. \end{array}$$

RETRACTED

### 2.4. Analysis of Emotional and Psychological State Recognition Method Based on Decision Layer Fusion

The emotional and psychological state recognition of facial expressions is mainly analyzed. One frame of facial expression image in each video image in the database is selected as a key frame for facial expression emotional state recognition. These samples are divided into the training, validation, and test sets. A ConvNet network is used to train a facial expression-based emotional and physiological state recognition model.  Figure 5 displays the ConvNet network architecture.

From Figure 5, the size of the original image input to the neural network is 32∗32. The number of training sets is limited. The input original image size is randomly cropped to 30∗30 each time to prevent overfitting, and these images are randomly flipped horizontally. The network structure is divided into four stages. The first stage consists of a convolutional layer, a max-pooling layer, and a local response normalization layer. The second stage consists of a convolutional layer, an average pooling layer, and a regional response normalization layer. The third stage consists of one convolutional layer and one intermediate pooling layer. The fourth stage is the classification stage, which consists of a fully connected layer and an output layer. The output layer realizes the mapping between the feature and the classification probability distribution through the Soft-Max function and outputs the probability distribution of the six emotional labels. The calculation formula is as follows; *x*_*i*_ represents the input test sample.

(3) $$\begin{array}{c} \rho_{fac,n}=\frac{\exp\left(x_{n}\right)}{\sum_{i=1}^{6}\exp\left(x_{i}\right)},n\epsilon \left\{1,2,\cdots ,6\right\}. \end{array}$$

### 2.5. Probit Models to Examine Emotional Design

This paper examines the analysis of personality traits based on an emotional and psychological state recognition scheme for herdsmen's credit behavior. The specific research is based on the identification of emotional and psychological states, the behavior analysis of herdsmen's demand for formal credit, availability of formal credit, and the amount of formal credit. Among them, the credit availability of herdsmen can be investigated in two stages. The first stage is whether the herdsmen obtain loans from formal financial institutions, usually represented by a zero to one dummy variable. The second stage is the quota received by farmers, which is generally expressed as a truncation variable greater than zero. Therefore, a Probit model is first constructed to test the influence of emotional and psychological states on herdsmen's formal credit demand and whether to obtain loans. The Probit model is demonstrated as

(4) $$\begin{array}{c} \mathrm{Pr}\left(Y_{i}^{*}=1\right)=\alpha_{0}+\alpha_{1}\;{\text{ope}}_{i}+\alpha_{2}\;{\text{con}}_{i}+\alpha_{3}\;{\mathrm{ext}}_{i}+\alpha_{4}\;{\text{agr}}_{i}+\alpha_{i}\;{\text{controls}}_{i}+\varepsilon_{i}. \end{array}$$

In Equation (4), *Y*_*i*_^∗^ is a dummy variable. *Y*_1_^∗^ = 1 means the herdsmen have formal credit needs. If it is not one, there is no formal credit need. The *controls* are control variables. *ε*_*i*_ is the residual term.

RETRACTED

Then, a Heckman two-stage model is constructed to examine the influence of the emotional and psychological state on herdsmen's formal credit line. The first stage is the Probit model, which describes the possibility of farmers obtaining formal credit. The second stage describes the material availability of credit, which is how much credit is available. “Have a credit rating” and “Have informal credit” are identification variables. The first-stage equation is used to calculate the Nimirs ratio. It is added to the second-stage model as a control variable. If its coefficient is significantly nonzero, the selection of the Heckman two-stage model is effective.

(5) $$\begin{array}{c} \mathrm{Pr}=\left(Y_{2}^{*}=1\right)=\beta_{0}+\beta_{1}\;{\text{ope}}_{i}+\beta_{2}\;{\text{con}}_{i}+\beta_{3}{\mathrm{ext}}_{i}+\beta_{4}\;{\text{agr}}_{i}+\beta_{i}\;{\text{controls}}_{i}+\mu_{i},\\ {\text{Y}}_{3}=\delta_{0}+\delta_{1}\;{\text{ope}}_{i}+\delta_{2}\;{\text{con}}_{i}+\delta_{3}{\mathrm{ext}}_{i}+\delta_{4}\;{\text{agr}}_{i}+\delta_{i}\;{\text{controls}}_{i}+\mu_{i}. \end{array}$$

Stratified random sampling is adopted here. The data comes from the research group's household survey of 200 farmers in three autonomous banners in XX District. The survey data is collected and organized, and the office software is used for scientific analysis and calculation of the collected data. The detailed information lays a solid foundation for the following research work. The questionnaire design adopted a multidimensional questionnaire. Each dimension contains three to six items, including one to four reverse scoring items. A total of 25 topics are designed around experience, cognition, practice, and active personality. The research is divided into two aspects. The first is the basic situation at the village level, the circulation of grasslands, and the economic environment. The second is the basic household information, pasture information, production and operation information, and credit insurance information at the household level.

RETRACTED

The reliability and validity of the questionnaire are analyzed. Reliability analysis is mainly used to measure whether the answer results of experimental samples are reliable. For example, the same object is measured multiple times. If the results of multiple measurements are close, the value of the result is considered credible. If the results of each measurement are different, the reliability is low. Validity analysis simply refers to the validity and accuracy of the questionnaire design. It is used to measure whether the design of the item is reasonable. Validity can be further divided into content validity, construct validity, and criterion validity. Content validity is usually a verbal description of the validity of the questionnaire. For example, references or authoritative sources are used to demonstrate the authority and validity of the questionnaire. Commonly used reliability coefficients include Cronbach's alpha coefficient, half coefficient, and sampling suitability measure Kaiser-Meyer-Olkin (KMO), which can be analyzed in the software Spssau. The value of the Cronbach's coefficient is 0.96 based on the reliability test of this questionnaire, and the half correlation coefficient is between 0.85 and 0.89, which shows that the reliability of the questionnaire is good. Based on the validity test, the KMO value reaches 0.92, indicating that the validity of the questionnaire is good.

The sampling method of the survey is stratified random sampling. First, pure animal husbandry counties (autonomous flags) within each city (league) are divided into high and low groups according to their gross domestic product considering regional differences and data availability. One county (autonomous banner) is randomly selected from each group. Second, each county (autonomous banner) is randomly selected from two to three sample townships. Finally, one to two sample villages are drawn from each township. Home interviews are used to fill out the questionnaires. A total of 200 questionnaires are collected in this survey. A total of 196 valid questionnaires are obtained after invalid questionnaires are excluded, with an effective rate of 98%.

In addition, the processing efficiency model using maximum likelihood estimation is selected to further study the influence of emotional and psychological positive state characteristics on farmers' formal credit behavior.

(6) $$\begin{array}{c} Y_{i}=\gamma_{0}+\gamma_{1}\;ope_{{\text{high}}_{1}}+\gamma_{i}W_{i}+\mu_{i},\\ T_{i}^{*}=\delta_{0}+\delta_{1}\;Z_{i}+\mu_{i}. \end{array}$$

RETRACTED

## 3. Results

### 3.1. Descriptive Statistical Results Analysis

The descriptive analysis of the respondents is shown in Figure 6.

From Figure 6, the demand for formal credit among the respondents is strong. One hundred twenty farmers have obtained loans from formal financial institutions, accounting for 61.1% of the farmers who need formal credit, indicating that the sample herdsmen have low availability of formal credit. This is consistent with the conclusion of the People's Bank of China's herdsmen's credit situation questionnaire survey and analysis team. In terms of the loan amount, the average loan amount of the sample farmers is 158,000 yuan, with a variance of 20.6. This shows that the demand for credit lines of the sample farmers is generally high, but the internal differences are also large. The average age of the interviewed farmers is 51.4 years old, and the overall age level is high, judging from the individual and family characteristics of the sample herdsmen. The average years of education are 7.2 years, corresponding to junior high school education. The overall level is low. The herdsmen are a family of four. The average annual household income is about 100,000 yuan per year. The per capita land size is approximately 1.54 mu. About 36.5% of rural households use mobile internet payment methods, indicating that the penetration of Internet finance is still low.

### 3.2. Regression Analysis Results

Regression analysis is carried out on the influence of the survey variables on the credit behavior of farmers, and the specific results are shown in Table 1.

From Table 1, the effects of open emotional psychology, conscientiousness psychology, and extroversion psychology on herdsmen's credit demand are statistically positive at 1%, 5%, and 1%, respectively. The marginal effects are 18.73%, 10.71%, and 15.96%, respectively. This implies that the probability of herdsmen generating credit demand increases by 18.73%, 10.71%, and 15.96%, respectively, for every one-unit increase in emotional psychology.

The link between the positive emotional state and herdsmen's credit behaviors is further analyzed. It is used as the standard to take the average of all sample values of positive emotional and psychological characteristics. The ones above the standard value are set as the sample group of high emotional and psychological characteristics. Besides, the sample groups are set as training groups, and the differences between the groups are analyzed. The results are revealed in Figure 7.

From Figure 7, the herdsmen with high scores of emotional and psychological characteristics have higher credit demand, credit availability, and credit line than herdsmen with low emotional and psychological characteristics. The difference between groups is significant, at least at the 10% significance level. Furthermore, there are substantial differences in other characteristics between the two groups of samples. This indicates that the distribution between the two groups of farmers is not completely random. An empirical analysis of credit behavior is conducted on herdsmen with high emotional and psychological characteristics, and the results are shown in Table 2.

RETRACTED

From Table 2, herdsmen with high emotional and psychological scores strongly demand credit and are likely to obtain credit. Specifically, the herdsmen with high emotional and psychological scores have a 71% higher probability of generating credit demand and a 33.47% higher likelihood of obtaining formal credit than those with low emotional and psychological scores. The regression results of the second stage of the Heckman model show that herdsmen with high emotional and psychological scores are more likely to obtain more extensive credit lines than herdsmen with low emotional and psychological scores. The difference between the two is about 40,400 yuan.

## 4. Conclusion

This paper studies the current herdsmen's credit behavior based on the emotional and psychological state identification scheme. A related identification research model is designed according to the current status of herdsmen's credit behavior and the action mechanism of the psychological identification program. The herdsmen's credit behavior is analyzed according to the survey data. The results show that herdsmen with high scores of emotional and psychological characteristics have strong demand for credit, are likely to obtain credit, and have high credit lines. Herdsmen with low scores of emotional and psychological characteristics have low or no obvious demand for credit, and their credit availability is also low. Moreover, the treatment effect model analyzes the influence of emotional and psychological characteristics scores on herdsmen's credit behavior. The study finds that herdsmen with high emotional and psychological characteristics have a 71% higher probability of generating credit demand than farmers with low openness. They are also 33.47% more likely to obtain credit than herdsmen with low emotional and psychological characteristics. They are also expected to obtain high loan amounts. The robustness test results indicate that the experimental results are in good agreement. The disadvantage is that the number of surveyed objects is relatively small, and the geographical area is limited. The research work on the key techniques of psychometrics done here has broad application prospects and practical significance. Although some achievements have been achieved, there is still a long way to go before the actual promotion and use. The follow-up research work can also be improved and perfected from the following aspects. Firstly, the universal intelligent psychological evaluation system can operate stably and reliably after systematic testing. This is in line with the expected demand design. Physiological and behavioral data of different groups can be easily collected through the promotion and use of the system. In the follow-up work, artificial intelligence algorithms such as deep learning can be added to the server to research various data aggregation and mining technologies. It will help build a group mental situational awareness model to serve all areas of society well.

RETRACTED

## Figures and Tables

**Figure 1:** Step diagram of emotional and psychological recognition.

**Figure 2:** Feature layer fusion process diagram.

**Figure 3:** The decision-making layer fusion process diagram.

**Figure 4:** The influence of emotional and psychological characteristics on herdsmen's credit behavior (a) direct influence; (b) indirect influence.

**Figure 5:** ConvNet network architecture diagram.

**Figure 6:** The detailed situation map of the investigated persons; (a) the credit behavior distribution map; (b) the identity map of the investigated persons.

**Figure 7:** Descriptive analysis of herdsmen with high scores on emotional and psychological characteristics (a) distribution map of credit behavior; (b) identity map of respondents.

**Table 1:** Regression analysis results.

	Demand	Availability	Amount	
Gender	0.0699 (0.10)	0.2024∗∗∗ (2.85)	0.0004 (0.00)	0.5153 (0.21)
Age	-0.0148∗∗∗ (-5.54)	0.0193∗∗∗ (-6.53)	-0.059 (-1.63)	-0.2215∗∗ (-2.17)
Edu	0.0489∗∗∗ (5.01)	0.0010 (0.92)	0.0115 (0.90)	0.4373 (1.30)
Family-number	0.0399∗∗ (2.46)	0.0585∗∗∗ (3.30)	0.0417∗ (1.94)	1.1561∗∗ (1.73)
Income	0.0021 (1.61)	0.0048∗∗ (3.40)	0.0038∗∗ (2.52)	0.0063 (1.01)
Land	-0.0096 (-0.52)	0.0474∗∗ (2.39)	0.0192 (0.77)	1.4094∗∗∗ (2.98)
Social	0.0045 (1.26)	0.00093∗∗ (2.46)	0.0091∗∗ (2.04)	0.0225 (0.21)
Odt			0.4371∗∗∗ (4.57)	
Crg			1.1607∗∗∗ (13.45)	
Constant term	0.1800	-1.3141∗∗∗	-2.0781∗∗∗	-6.5206
	(0.53)	(-3.51)	(-4.67)	(0.54)
*γ*			-8.3054∗∗∗	

**Table 2:** Graph of regression analysis results.

Regression analysis	Residual covariance			Residual correlation		
	Amount	Availability	Demand	Amount	Availability	Demand
	0.9385	0.7394	0.6282	0.4373	0.8567	0.6557
	Wald chi2			Emotional psychological characteristics		
	Amount	Availability	Demand	Amount	Availability	Demand
	34.69	20.06	86.22	0.1808	0.1672	0.1873

RETRACTED

## Data Availability

The data used to support the findings of this study are included within the article.
